The article "The Impact of Noninvasive Ventilator Assisted Ventilation Nursing Combined with Mechanical Vibration on the Level of Heart Failure Indexes in ICU Patients with Acute Heart Failure" was retracted in 2023. Reasons: signs of a paper mill; suspected computer-generated content; unreliable results or conclusions; concerns about the data.

# The Impact of Noninvasive Ventilator Assisted Ventilation Nursing Combined with Mechanical Vibration on the Level of Heart Failure Indexes in ICU Patients with Acute Heart Failure

**DOI:** 10.1155/2022/7234357

**Published:** 2022-02-26

**Authors:** Wenze Li, Qifeng Lou

**Affiliations:** ^1^Tongde Hospital of Zhejiang Province, Hangzhou 310012, China; ^2^Affiliated Hangzhou First People's Hospital, Zhejiang University School of Medicine, Hangzhou 310012, China

## Abstract

The acute attack of acute heart failure or the continuous deterioration of cardiac function leads to a series of changes such as reduced cardiac contractility, increased cardiac load, and a sudden drop of acute cardiac output, which eventually cause pulmonary circulation congestion and acute dyspnea due to acute pulmonary congestion. To observe the impact of noninvasive ventilator-assisted ventilation nursing combined with mechanical vibration on the level of heart failure indexes in intensive care unit (ICU) patients with acute heart failure, 120 patients with acute heart failure who were treated in the ICU ward of our hospital from September 2018 to March 2021 were selected, and the qualified subjects were divided into two groups according to the 1 : 1 principle by a simple random method. 120 patients were given conventional symptomatic treatment and noninvasive ventilator-assisted ventilation. The control group received conventional nursing intervention, and the observation group was given noninvasive ventilator-assisted ventilation nursing and mechanical vibration intervention. The respiratory system indexes, heart rate, blood pressure, central venous pressure, N-terminal B-type natriuretic peptide precursor (NT-proBNP), cardiac troponin *T* (cTnT), and cardiac function indexes of the two groups of patients are recorded, and the prognosis of the two groups is compared. After intervention, the partial pressure of oxygen (PaO2) and blood oxygen saturation (SpO2) in the two groups were higher than those before intervention, while the partial pressure of carbon dioxide (PaCO2), respiration (RR), heart rate, blood pressure, and central venous pressure were lower than those before intervention (*P* < 0.05). Compared with the control group, PaO2, SpO2, systolic blood pressure, diastolic blood pressure, and central venous pressure of the observation group after intervention were significantly higher, while PaCO2, RR, and heart rate were significantly lower (*P* < 0.05). Compared with the control group, the LVEF of the observation group after intervention was significantly higher, while NT-proBNP, cTnT, LVESD, and LVEDD were markedly lower (*P* < 0.05). The ventilation time and ICU hospitalization time in the observation group were shorter than those in the control group, and the pulmonary infection rate was lower than in the control group. The remission time of infection in patients with pulmonary infection was shorter than that in the control group. When comparing the 28d mortality rate with the control group, the difference was not statistically significant (*P* > 0.05). Noninvasive ventilator-assisted ventilation nursing combined with mechanical vibration can improve hypoxemia symptoms and heart function, stabilize hemodynamics, shorten the course of disease and reduce the occurrence of lung infections for those patients with acute heart failure in the ICU.

The article "The Impact of Noninvasive Ventilator Assisted Ventilation Nursing Combined with Mechanical Vibration on the Level of Heart Failure Indexes in ICU Patients with Acute Heart Failure" was retracted in 2023. Reasons: signs of a paper mill; suspected computer-generated content; unreliable results or conclusions; concerns about the data.

## 1. Introduction

Acute heart failure is one of the common acute coronary syndromes in clinical practice. Under the influence of various reasons, the cardiac structure or function is abnormal, which suddenly causes some syndromes characterized by pulmonary edema, pulmonary congestion, and systemic congestion, in addition to low perfusion of tissues and organs. Without timely treatment, the mortality rate is higher [1]. The intensive care unit (ICU) is an important place for the treatment of patients with acute heart failure. Comprehensive treatments such as cardiotonic, diuretic, vasodilator, noninvasive ventilator-assisted ventilation can play an effective role in their treatment. Among these methods, the noninvasive ventilator is essential to improve the myocardial blood supply and ejection fraction of patients. In addition, the quality of nursing work in the treatment process exerts an important impact on the prognosis of patients [2].

Ventilator-associated pneumonia is prone to occur during the use of noninvasive ventilators, resulting in increased airway secretions, while patients with acute heart failure in the ICU have a weak ability of autonomous expectoration [3]. Mechanical vibration expectoration uses the knocking effect of the machine to help loosen and discharge sputum on the surface of the airway mucosa to improve lung ventilation [4]. In order to optimize the prognosis of patients with acute heart failure in ICU, this study used noninvasive ventilator-assisted ventilation nursing combined with mechanical vibration to treat patients with acute heart failure in ICU and observed its impact on the level of heart failure indicators. The report is further discussed in this study.

## 2. Data and Methods

### 2.1. General Information

120 patients with acute heart failure treated in the ICU ward of our hospital from September 2018 to March 2021 were selected. This study was approved by the hospital ethics committee.

The inclusion criteria are as follows: (1) according to the standard of acute heart failure in China's Emergency Clinical Practice Guidelines for Acute Heart Failure (2017) [5] , patients should be diagnosed by electrocardiogram, chest X-ray, and echocardiography; (2) age ≥60 years, ≤ 80 years; (3) with hypoxemia (SpO2 < 90% or PaO2 < 60 mmHg) and left ventricular ejection fraction (LVEF) < 40%; (4) cardiac functional grade III ∼ IV; and (5) patients' informed consent.

The article "The Impact of Noninvasive Ventilator Assisted Ventilation Nursing Combined with Mechanical Vibration on the Level of Heart Failure Indexes in ICU Patients with Acute Heart Failure" was retracted in 2023. Reasons: signs of a paper mill; suspected computer-generated content; unreliable results or conclusions; concerns about the data.

The exclusion criteria are as follows: (1) Glasgow Coma Scale score ≤12; (2) accompanied with pneumothorax, type II respiratory failure, pulmonary embolism, and other serious lung diseases; (3) uncontrolled severe arrhythmia or chest trauma; (4) accompanied with severe cerebrovascular disease, or coronary angiography or interventional therapy during hospitalization; (5) accompanied with severe hematopoietic and immune system diseases; and (6) accompanied with malignant tumors and mental illness. 120 patients were randomly divided into two groups according to the principle of 1 : 1. Comparing the general data of the two patient groups, the difference was not statistically significant (*P* > 0.05).  Table 1 shows the comparison of general data between the two patient groups.

## 3. Method

All patients were given conventional symptomatic treatment and noninvasive ventilator-assisted ventilation. They were given adequate rest, low salt and fat in addition to the water-limited diet. Furthermore, they were given high-flow oxygen inhalation, cardiotonic, diuretic, vasodilator, and other medications. Heart failure-inducing factors such as infection, arrhythmia, excessive physical consumption, emotional excitement, moderate-to-severe anemia, renal damage, and improper intravenous infusion should be actively removed. The noninvasive ventilator was Weinmann bilevel positive pressure noninvasive ventilator from Germany Vanman Company. The ventilation mode was S/T and the ventilator parameters were IPAP 12–16 cm H2O, EPAP4–8 cm H2O, oxygen flow rate 4–6 L/min, and respiratory rate 12–20 times/min.

The control group was given routine nursing intervention. During the treatment, vital signs such as blood pressure, heart rate, and body temperature were closely monitored, and skin color and mental state were also observed. Noninvasive ventilators should be used strictly in accordance with the operating rules, and the ventilator parameters should be timely adjusted according to the blood gas analysis index and respiratory index of patients. Venous access should be established and medication given according to doctor's advice. Prepare rescue equipment and drugs, regularly help patients turn over and buckle back, and cooperate with doctors to clean up respiratory secretions when necessary.

The article "The Impact of Noninvasive Ventilator Assisted Ventilation Nursing Combined with Mechanical Vibration on the Level of Heart Failure Indexes in ICU Patients with Acute Heart Failure" was retracted in 2023. Reasons: signs of a paper mill; suspected computer-generated content; unreliable results or conclusions; concerns about the data.

The observation group was given noninvasive ventilator-assisted ventilation nursing and mechanical vibration intervention. Noninvasive ventilator should be used strictly in accordance with the operating rules, and the ventilator parameters should be adjusted according to the blood gas analysis index and respiratory index of patients. Pay attention to the observation of patients with gastric distension, nasal injury, upper gastrointestinal reflux, and other complications. Guide patients to use the ventilator correctly, try to breathe through nose, avoid breathing through mouth, and remove ventilator when eating. Regularly check the air tightness of the mask in order to avoid conjunctivitis and ventilator compensation due to air leakage. Before the use of noninvasive ventilators, the skin of patients was scored. During the use of a noninvasive ventilator, the mask was loosened properly, the tight band of the mask was adjusted, the gauze was filled when necessary, and the compressed skin was massaged regularly to prevent nasal and facial pressure sores. Noninvasive ventilation treatment should be avoided immediately after full meals, and noninvasive respiration should be performed at least 1h after meals to help patients maintain a 30–40° semirecumbent position to prevent reflux and aspiration caused by increased abdominal pressure. The multiple-frequency vibration expectoration machine of Weihai Bohua Medical Equipment Co., Ltd. was regularly used for mechanical vibration expectoration. The patients were in lateral position with an initial frequency of 15–30 cps, 10–20 min/time. After one side was completed, the patients were assisted to turn over and knock on the other side 2–4 times/min, 1–2 h before or 2 h after eating.

### 3.1. Detection Method

The respiratory system indexes, heart rate, blood pressure, central venous pressure, N-terminal pro-B-type natriuretic peptide (NT-proBNP), cardiac troponin *T* (cTnT), and cardiac function indexes of the two groups before and after intervention were recorded. Blood gas analysis was performed on the radial artery blood of patients before and after the intervention. In addition, the levels of oxygen partial pressure (PaO2), oxygen saturation (SpO2), and carbon dioxide partial pressure (PaCO2) were detected. The detection instrument was the Danish ABL90 blood gas analyzer. The respiratory (RR), heart rate, blood pressure, central venous pressure, and other indicators in the PC-9000B ECG monitor were recorded. Left ventricular ejection fraction (LVEF), left ventricular end-systolic diameter (LVESD), and left ventricular end-diastolic diameter (LVEDD) were detected by ultrasound before and after intervention in the two groups. The detection instrument used was the Philips IE33 color Doppler ultrasound diagnostic instrument, and the probe frequency was 3.5–7.5 MHz. 2 ml fasting venous blood samples were taken before and after the intervention, placed in an EDTA anticoagulant tube, then centrifuged 1h after blood collection at 4000r/min for 10 min. Serum NT-proBNP and cTnT were detected by an enzyme-linked immunosorbent assay kit (Shanghai enzyme-linked biotech Co., Ltd.) and an electrochemiluminescence method (Shanghai enzyme-linked biotech Co., Ltd.), respectively. Detection instrument: Shenzhen Mairui Medical Electronics Co., Ltd. RT-96 A enzyme-labeled instrument.

The article "The Impact of Noninvasive Ventilator Assisted Ventilation Nursing Combined with Mechanical Vibration on the Level of Heart Failure Indexes in ICU Patients with Acute Heart Failure" was retracted in 2023. Reasons: signs of a paper mill; suspected computer-generated content; unreliable results or conclusions; concerns about the data.

### 3.2. Statistical Methods

The data were processed by SPSS19.0, and the enumeration data conforming to the normal distribution were described by ($\bar{\chi }$ ± *s*). The *t*-test was used for comparison, and the enumeration data were described by the number of cases (percentage). The *χ*^2^ test was used for comparison, which had statistical significance (*P* < 0.05).

## 4. Experimental Results

### 4.1. Comparison of Respiratory Indicators between the Two Groups

Before intervention, compared with the respiratory indicators between the two groups, the difference was not statistically significant (*P* > 0.05). After intervention, PaO2 and SpO2 in both groups increased compared with preintervention, while PaCO2 and RR decreased compared with preintervention (*P* < 0.05). Compared with the control group, PaO2 and SpO2 were significantly higher in the observation group after intervention, while PaCO2 and RR were lower (*P* < 0.05).  Table 2 shows the comparison of the two groups of respiratory indicators.

### 4.2. Comparison of Heart Rate, Blood Pressure, and Central Venous Pressure between the Two Groups

Before intervention, heart rate, blood pressure, and central venous pressure were compared between the two groups, and the difference was not statistically significant (*P* > 0.05). After intervention, heart rate, blood pressure, and central venous pressure were lower than those before intervention (*P*< 0.05). The systolic pressure, diastolic pressure, and central venous pressure were significantly higher in the observation group after intervention, while the heart rate was lower, compared with the control group (*P* < 0.05).  Table 3 shows the comparison of heart rate, blood pressure, and central venous pressure in the two groups.

### 4.3. Comparison of NT-proBNP, cTnT, and Cardiac Function Indicators between the Two Groups

Before intervention, compared with the NT-proBNP, cTnT, and cardiac function indicators between the groups, the difference was not statistically significant (*P* > 0.05). After intervention, LVEF in both groups was higher than that before intervention, while NT-proBNP, cTnT, LVESD, and LVEDD were lower than those before intervention (*P* < 0.05). LVEF was markedly higher in the observation group after intervention, while the NT-proBNP, cTnT, LVESD, and LVEDD were lower, compared with the control group (*P* < 0.05).  Table 4 shows the comparison of the two groups of NT-proBNP, cTnT, and cardiac function indicators.

The article "The Impact of Noninvasive Ventilator Assisted Ventilation Nursing Combined with Mechanical Vibration on the Level of Heart Failure Indexes in ICU Patients with Acute Heart Failure" was retracted in 2023. Reasons: signs of a paper mill; suspected computer-generated content; unreliable results or conclusions; concerns about the data.

### 4.4. Comparison of the Prognosis between the Two Groups

The ventilation time and ICU hospitalization time in the observation group were shorter than those in the control group, the pulmonary infection rate was lower than that in the control group, and the remission time of infection in patients with pulmonary infection was shorter than in the control group. 28d mortality was compared with the control group, and the difference was not statistically significant (*P* > 0.05).  Table 5 shows the comparison of the two groups.

## 5. Experimental Data Analysis

Acute heart failure is a complex syndrome with clinical manifestations of dyspnea and even respiratory failure, which is characterized by a sudden onset and high mortality, and is one of the important causes of death in ICU patients [6]. In addition to conventional cardiac, diuretic, vasodilator drug treatment, and mechanical ventilation can improve respiratory function, which is widely used in the treatment of acute heart failure [7]. However, mechanical ventilation may cause ventilator-associated pneumonia and further affect ventilation function. Therefore, nursing work in the treatment of ICU patients with acute heart failure should be highly valued and actively prevent and treat various mechanical ventilation-related complications in order to improve the prognosis of patients [8]. Mechanical vibration expectoration is a commonly used treatment method for respiratory diseases, which can accelerate expectoration by promoting airway mucus relaxation, liquefaction, strengthening cilia oscillation, and improving pulmonary congestion and systemic circulation congestion through mechanical percussion. It has been applied in the treatment of severe pneumonia, chronic obstructive pulmonary disease, elderly chronic bronchitis, and postoperation [9], and so forth.

Nursing intervention in the process of noninvasive ventilator-assisted ventilation is of great significance to improve the effect of assisted ventilation and reduce complications. In this study, it was found that noninvasive ventilator-assisted ventilation nursing combined with mechanical vibration can improve the symptoms of hypoxemia in patients with acute heart failure in the ICU, promote respiratory function, and help increase heart rate, blood pressure, and central venous pressure by detecting PaO2, SpO2, PaCO2, RR, and other indicators before and after intervention in the two groups. This is because the nursing intervention in the process of noninvasive ventilator-assisted ventilation prevents gastric distension by guiding patients to correctly cooperate with the use of ventilators, trying to breathe through the nose, removing ventilators when eating, and regularly checking the air tightness of masks. During the use of noninvasive ventilators, measures such as proper adjustment of the mask, filling of gauze, and regular massage of compressed skin were taken to prevent nasal and facial pressure ulcers. Helping patients take 30–40° semirecumbent positions and avoiding a full meal immediately afterward without invasive ventilation and other measures to prevent reflux and aspiration. Mechanical vibration expectoration is used in small and medium airways by mechanical force to promote plasma cell secretion and dilute sputum, relax secretions and strengthen cilia movement to accelerate expectoration. Knock can also accelerate local lymphatic reflux, reduce pulmonary edema, and lower pulmonary ventilation resistance. Improvement of pulmonary ventilation function can increase oxygen supply, promote carbon dioxide emissions, and improve blood gas analysis results [10, 11].

The article "The Impact of Noninvasive Ventilator Assisted Ventilation Nursing Combined with Mechanical Vibration on the Level of Heart Failure Indexes in ICU Patients with Acute Heart Failure" was retracted in 2023. Reasons: signs of a paper mill; suspected computer-generated content; unreliable results or conclusions; concerns about the data.

LVEF, LVESD, and LVEDD are important indicators reflecting cardiac pumping function. The slump in LVEF and the increase in LVESD and LVEDD for patients with acute heart failure, which cannot effectively pump blood and meet the needs of organs [12]. Under normal circumstances, serum NT-proBNP and cTnT levels are extremely low, which are extensively released into the blood after mechanical injury of ventricular myocytes, leading to an increase of serum NT-proBNP and cTnT levels [13, 14]. In this study, LVEF, LVESD, LVEDD, and serum NT-proBNP and cTnT levels were detected by ultrasound, which found that noninvasive ventilator-assisted ventilation nursing combined with mechanical vibration can improve cardiac function in patients with acute heart failure in the ICU. This is due to mechanical vibration expectoration which helps promote the discharge of airway secretions, relieve bronchospasm, eliminate edema, reduce pulmonary ventilation resistance, increase blood oxygen concentration, make myocardial blood supply increase, and decrease the release of NT-proBNP and cTnT caused by myocardial ischemia and hypoxia injury [15–17].

This study also found that noninvasive ventilator-assisted ventilation nursing combined with mechanical vibration could shorten the ventilation time and ICU hospitalization time of patients with acute heart failure in the ICU, reduce the pulmonary infection rate, and shorten the infection remission time of patients with pulmonary infection [18–22]. This is because the frequency of mechanical vibration is similar to the natural physiological frequency of the human body, which can effectively promote the discharge of sputum, reduce the accumulation of sputum in the airway, and thus lighten the load of local pathogens in the airway, which is conducive to the prevention of pulmonary infection and the promotion of rehabilitation of patients. But the difference of 28d mortality between the two groups was not statistically significant. This is because the occurrence of death is related to multiple factors such as primary disease, complications, and patient constitution. In future clinical work, large sample studies should be accumulated to analyze the impact of noninvasive ventilator-assisted ventilation nursing combined with mechanical vibration on the mortality risk of ICU patients with acute heart failure.

The article "The Impact of Noninvasive Ventilator Assisted Ventilation Nursing Combined with Mechanical Vibration on the Level of Heart Failure Indexes in ICU Patients with Acute Heart Failure" was retracted in 2023. Reasons: signs of a paper mill; suspected computer-generated content; unreliable results or conclusions; concerns about the data.

## 6. Conclusion

In order to observe the impact of noninvasive ventilator-assisted ventilation nursing combined with mechanical vibration on the level of heart failure indexes in intensive care unit (ICU) patients with acute heart failure, 120 patients with acute heart failure who were treated in the ICU ward of our hospital from September 2018 to March 2021 were selected, and the qualified subjects were divided into two groups according to the 1 : 1 principle by a simple random method. The experimental results show that noninvasive ventilator-assisted ventilation nursing combined with mechanical vibration can improve the symptoms of hypoxemia and cardiac function in patients with acute heart failure in the ICU, stabilize hemodynamics, shorten the course of disease, and reduce the incidence of pulmonary infection.

## Figures and Tables

**Table 1:** Comparison of general data between the two patient groups.

General information		Treatment group (*n* = 60)	Experimental group(*n* = 60)
Gender (*n*)	Male	33 (55.00)	35 (58.33)
	Female	27 (45.00)	25 (41.67)

Age (years)		70.14 ± 4.52	69.89 ± 5.01
LVEF (%)		35.14 ± 3.56	34.98 ± 3.85

BMI (kg/m^2^)	<18.5 (lean)	12 (20.00)	10 (16.67)
	18.5～24.9 (normal)	31 (51.67)	29 (48.33)
	>25 (overweight)	17 (28.33)	21 (35.00)

Cardiac functional grading (*n*)	III	37 (61.67)	35 (58.33)
	IV	23 (38.33)	25 (41.67)

Academic (*n*)	Junior high school and below	14 (23.33)	18 (30.00)
	Secondary and high schools	25 (41.67)	22 (36.67)
	College or higher	21 (35.00)	20 (33.33)

Underlying diseases (*n*)	Valve heart disease	24 (40.00)	21 (35.00)
	Ischemic heart disease	17 (28.33)	18 (30.00)
	Hypertensive heart disease	10 (16.67)	11 (18.33)
	Dilated cardiomyopathy	9 (15.00)	10 (16.67)

Note: BMI is the body mass index.

The article "The Impact of Noninvasive Ventilator Assisted Ventilation Nursing Combined with Mechanical Vibration on the Level of Heart Failure Indexes in ICU Patients with Acute Heart Failure" was retracted in 2023. Reasons: signs of a paper mill; suspected computer-generated content; unreliable results or conclusions; concerns about the data.

**Table 2:** Comparison of the two groups of respiratory indicators ($\bar{\chi }$ ± *s*).

Index	Treatment group (*n* = 60)		Experimental group (*n* = 60)	
	Before intervention	Postintervention	Before intervention	Postintervention
PaO2 (mmHg)	48.58 ± 8.11	59.63 ± 6.85①	19.05 ± 7.53	68.25 ± 5.81①②
PaCO2 (mmHg)	72.01 ± 5.88	52.12 ± 4.61①	70.98 ± 6.04	42.11 ± 4.08①②
SpO2 (%)	75.85 ± 4.85	86.96 ± 4.01①	74.98 ± 4.96	94.78 ± 3.11①②
RR (times/min)	30.12 ± 3.05	21.55 ± 2.51①	29.89 ± 3.24	18.85 ± 1.74①②

Note: *P* < 0.05 was compared before intervention with this group, and *P* < 0.05 was compared with the control group.

**Table 3:** Comparison of heart rate, blood pressure, and central venous pressure in the two groups ($\bar{\chi }$ ± *s*).

Index	Treatment group (*n* = 60)		Experimental group (*n* = 60)	
	Before intervention	Postintervention	Before intervention	Postintervention
Heart rate (times/min)	119.85 ± 12.41	101.11 ± 10.25①	121.14 ± 11.52	89.52 ± 8.14①②
Systolic pressure (mmHg)	125.01 ± 3.45	104.12 ± 3.95①	124.94 ± 3.85	116.05 ± 4.11①②
Systolic pressure (mmHg)	78.69 ± 5.11	62.85 ± 4.11①	78.41 ± 4.95	68.18 ± 4.13①②
Central venous pressure (mmHg)	15.45 ± 2.52	8.14 ± 1.41①	15.48 ± 2.49	9.41 ± 1.29①②

Note: *P* < 0.05 was compared before intervention with this group, and *P* < 0.05 was compared with the control group.

**Table 4:** Comparison of the two groups of NT-proBNP, cTnT, and cardiac function indicators ($\bar{\chi }$ ± *s*).

Index	Treatment group (*n* = 60)		Experimental group (*n* = 60)	
	Before intervention	Postintervention	Before intervention	Postintervention
NT-proBNP (pg/mL)	4597.25 ± 1024.32	2145.36 ± 751.02①	4614.01 ± 987.52	1687.25 ± 589.66①②
cTnT (pg/mL)	102.25 ± 8.05	81.45 ± 6.89②	101.89 ± 6.74	70.58 ± 5.14①②
LVEF (%)	35.14 ± 3.56	42.52 ± 3.96①	34.98 ± 3.85	48.96 ± 4.57①②
LVESD (mm)	42.36 ± 4.17	38.89 ± 3.54①	42.43 ± 3.95	34.51 ± 3.11①②
LVEDD (mm)	52.36 ± 5.98	49.74 ± 3.74①	52.24 ± 6.08	46.11 ± 3.21①②

Note: *P* < 0.05 was compared before intervention with this group, and *P* < 0.05 was compared with the control group.

**Table 5:** Comparison of the two groups.

Prognostic condition		Treatment group (*n* = 60)	Experimental group (*n* = 60)
Duration of ventilation (h)		78.96 ± 12.96	72.14 ± 10.05②
ICU hospital stay (d)		12.88 ± 3.25	10.74 ± 2.14②
Lung infection	Incidence (%)	7 (11.67)	1 (1.67)②
	Infection remission time (d)	5.14 ± 1.11	3.58 ± 0.78②
28d death rate		13 (21.67)	6 (10.00)

Note: *P* < 0.05 was compared with the controls.

## Data Availability

The simulation experiment data used to support the findings of this study are available from the corresponding author upon request.
